The article "Home language use and shift in Australia: Trends in the new millennium" was published in 2023. Journal: Front Psychol.

# Home language use and shift in Australia: Trends in the new millennium

**DOI:** 10.3389/fpsyg.2023.1096147

**Published:** 2023-02-09

**Authors:** Lubei Zhang, Linda Tsung, Xian Qi

**Affiliations:** ^1^School of foreign languages, Southwest Jiaotong University, Chengdu, China; ^2^School of languages and cultures, the University of Sydney, Darlington, NSW, Australia

**Keywords:** Australia, home language, language shift, multilingualism, multiculturalism

## Abstract

The 25 million Australians today are identified with more than 300 ancestries. People’s home language use and shift patterns had demonstrated great variations as more immigrants from Asia-Pacific regions entered Australia. The ethnolinguistic composition of Australia’s population had undergone substantial changes in the last few decades. Based on the statistics from Australian censuses, the present paper aims to analyze the changes of people’s home language use and the shift patterns in the new Millennium. Five sets of census data released by Australian Bureau of Statistics were adopted as the secondary data source and descriptive analysis was conducted to disclose the dynamic picture of different home languages in Australia after 2000. The results suggest that the number of home language speakers in Australia has soared up quickly in the last two decades and great variations have been found between the traditional European migrant groups and the newly Asian arrivers. Mandarin has overtaken Italian and Greek to become the most populous home language other than English used in Australia since 2011 and great regional differences were also found to exist among different states and territories. Moreover, the ranking order of different home language speakers had changed considerably as compared with that in the last century. The language shift rates of different language communities and their cross-tabulations with generations, gender, age, and duration of residence in the latest available censuses after 2000 also revealed diverse developmental directions. The findings give us a glimpse of the current status of different home languages in Australia and help us to identify the potential factors impacting the shifting trends of different language communities. A better understanding of the language needs of different migrant communities may further help policymakers set more effective plans to accommodate an increasingly diverse Australian society.

## 1. Introduction

With rich indigenous cultures and experience of mass immigration, Australia has long been taken as one of the world’s most multilingual and multicultural society (Burnley, 2001; Arvanitis et al., 2014; Bouma, 2016). The 25 million Australians today, identified with more than 300 ancestries, speak around 490 languages and observe a wide variety of cultural and religious traditions (ABS, 2021, 2022). About 22.3% of Australians today have reported to use another dominant language in their homes (ABS, 2021), which indicates a higher proportion of second language use in their professional, personal and social life. For decades, the language and cultural maintenance patterns of various migrant groups were under investigation by many linguists and sociologists (Clyne, 1991; Kipp et al., 1995; Clyne and Kipp, 1999; Smolicz et al., 2001; Perera, 2015), with the research focus mainly casted on the urban centers of Australia, such as Sydney and Melbourne. Immigration policies in different historical phases and the official language policies beheld by the Australian government have always been taken as a major factor affecting the language maintenance trends of different migrant groups. As Kalantzis et al. (1989) once commented that the position and survival of languages within a multicultural society were closely associated with power relations, self-determination, and access. In Australia, a policy of multiculturalism was claimed to be in operation since the early 1970s. Efforts have been made to encourage non-English speaking background (NESB) migrant groups to form state and national associations to maintain their cultures and to promote the survival of their community languages and heritage (Department of Immigration and Citizenship, 2007). After examining the linguistic situation in Sydney and Melbourne, Clyne et al. (2008) had characterized Australia as an increasingly multilingual nation. However, some other researchers argued that this was only true for languages of the recently arrived migrants (Forrest et al., 2020). A high percentage of language shift rates had been observed among those from most European origins. With a steady increase in the number of people born overseas across the whole country, especially in the neighboring Asia-Pacific regions, the ethnolinguistic demography of Australia has undergone substantial changes in recent years. What is the most recent picture regarding different migrant groups’ language shift patterns? Did they follow any rules? And are there any regional differences across the whole country? All these questions aroused our interests. The following sections, based on the most recent census statistics, will try to capture the dynamic picture of the immigrants’ language use patterns in home and their language shift trends after entering the new Millennium.

The article "Home language use and shift in Australia: Trends in the new millennium" was published in 2023. Journal: Front Psychol.

## 2. Literature review

Studies on the issues relating to linguistic maintenance of major migrant groups and their English proficiency in Australia have been conducted by many researchers based on the quinquennial census data. Research revealed that the rate of population speaking a language other than English (LOTE) at home had embodied the changes in Australia’s immigration policy on source countries and the absolute numbers of immigrants admitted by Australia annually. Most European languages brought by the early immigrants in the 1950s and 1960s were now in decline, exhibiting a high level of linguistic shift among their second generation. More than 90% of them had undergone linguistic shift by the second generation (Forrest and Dandy, 2017). However, significant variations were also found in different migrant communities (Clyne and Kipp, 2006). Greeks and those from the former Yugoslavia were exceptions (Forrest et al., 2020), with both of their first and second generations demonstrating a relatively lower language shift rates as compared with those from other European origins. On the other side, the surging of the immigrants from Middle Eastern and Asian countries in recent years had led to the booming of speakers of Mandarin Chinese, Arabic, Tagalog, Hindi, etc., some of which had already overtaken the traditional top community languages from Europe. Overall, as a result of Australia’s multicultural policy, the number of people speaking a LOTE at home in Australia has continued to increase and the origins of the home languages are more diversified.

The intergenerational language shift of different migrant groups is another research focus in recent years. The results had also demonstrated a very complex picture. It is widely acknowledged that the language shift was obvious in Australian-born generation, whose language shift rate was invariably higher than that in the first-generation migrants (Clyne and Kipp, 1996, 1997, 2006). The reason had always been attributed to the fact that the latter-generation migrants may not have a strong sense of cultural identity as their predecessors (Ngan and Chan, 2012; Li, 2017, 2018; Shen and Jiang, 2021). However, on the other hand, in most cases, the ranking order of the language shift rates of the second generation and the first generation were the same (Clyne and Kipp, 1997, 2006). In general, most European ancestry groups had experienced a higher intergenerational language shift than those from non-European countries, with the former exhibiting approximately 20% higher intergenerational shifting than the latter (Forrest et al., 2020). For the non-European background groups, research had also found a consistent and substantial difference between those whose mother was born overseas and father born in Australia and those whose father was born overseas and mother in Australia. When the mother was Australian-born, the language shift was usually much higher (Clyne and Kipp, 1996). As family remains for most migrant groups and their younger generations the main domain for heritage language use (Et-Bozkurt and Yağmur, 2022, p. 821), the influence of the marriage patterns and family language policies adopted by the migrant family on LOTE maintenance and shift cannot be neglected. In families with endogamous parents, the shift to English was generally lower than that in the intermarriage families, since the English contact within those families are limited (Clyne and Kipp, 1996). Other studies also found that the presence of grandparents in home, and parental perception of support from the educational environment on children’s linguistic orientation, etc. were all significant factors influencing the later generation’s language maintenance and shift. In all, great variations of language shift rates had been found to exist in the second-generation migrants. Those who were from Turkey, China, and Spain were setting at the lower end (Clyne and Kipp, 1996).

The article "Home language use and shift in Australia: Trends in the new millennium" was published in 2023. Journal: Front Psychol.

In addition, other social factors associated with the fluctuation of language shift rate also raised many scholars’ attention. Karidakis and Arunachalam (2016) analyzed the language shift rate of migrants based on the data from Australian 2011 Census. The results revealed that the language shift rate is inseparable from migrants’ gender, age, duration of residence, level of education, etc., and even within the same generation, the language shift to English varied much due to a variety of reasons. Generally, it is related to the size and concentration of the migrant groups (Vervoort et al., 2012), cultural distance from the mainstream (Clyne and Kipp, 1997, 2006), the religious beliefs and education level of the migrants (Smolicz, 1981; Fishman, 1997; Rubino, 2007; Perera, 2015, 2016), the family language policies adopted by the migrant family (Et-Bozkurt and Yağmur, 2022), the length of residence in Australia (Karidakis and Arunachalam, 2016), as well as other sociolinguistic and political factors (Smolicz, 1981; Mejia, 2015). Besides, homeland factors were also found to exert certain impacts. Perera (2015) asserted that one’s experience with English in the homeland, their sense of nationalism, as well as their devout faith in the ethnic religions would all support the preservation of a heritage language. Other factors, such as the development of traffic tools, the access to social media, such as Facebook and Instagram, and the infrastructure in migrant communities, the economic situation back in home countries had all exerted significant impacts on migrants’ language maintenance and shift (Karidakis and Arunachalam, 2016; Et-Bozkurt and Yağmur, 2022).

The article "Home language use and shift in Australia: Trends in the new millennium" was published in 2023. Journal: Front Psychol.

Although a number of studies had investigated these migrants’ language maintenance and shift trends in Australia, most of them were conducted based on the census data up to 2011 (Clyne and Kipp, 1997, 2006; Karidakis and Arunachalam, 2016; Forrest and Dandy, 2017). And only a few of them analyzed language maintenance and shift from a diachronic perspective and extend the research scope beyond the two major cities. Critical comparisons need to be done to identify the difference between the previous data period and the data since 2011.

## 3. The present study

Based on the data elicited from the previous five national censuses (2001, 2006, 2011, 2016, and 2021), this study aims to explore and analyze the changing trends of people’s home language use and shift patterns after the new millennium. Comparisons will be made across the generations, age groups, genders, residence durations, ancestries, as well as different inhabiting regions. The specific research questions are as follows:

1. What is the changing trend of the population speaking a LOTE at home during the past two decades? Are there any regional differences among eight administrative States and Territories?
2. What are the dynamic pictures of the language shift trend for the first-generation and second-generation migrants in Australia?

## 4. Method

### 4.1. Data

This paper is based on the data provided by the last five census statistics released by Australian Bureau of Statistics (ABS). The five data streams were chosen in order to represent a whole picture of people’s home language use patterns and the changing trends across the past two decades. As Australia’s national statistical agency, ABS carries out the Census of Population and Housing every 5 years, which covers a wide range of statistics, including the economic, social, and cultural makeup of Australia. Questions regarding people’s age, country of birth, religion, ancestry, language used at home, etc. were all listed in the census forms. It is believed to be the most comprehensive snapshot of the Australian society, reflecting the diversity of Australia by counting everyone (ABS, 2016b). As an authoritative source, the census data was thus adopted as secondary data for the present study.

According to the Australian Standard Classification of Languages (ASCL) 2016, four language variables have been identified, namely, first language spoken, language spoken at home, main language spoken, and main language other than English spoken at home. The data for this study were derived from the question on people’s “language spoken at home,” which was mainly designed to find out which languages other than English are spoken by people at home (ABS, 2016a). Since the question only allows for one answer, the number of response “English” does not represent all people speaking English, but those who only speak English. And if more than one other language had been used, only the one that had been used most frequently was recorded. Respondents’ language use in the homes of parents, relatives, or friends, or in community settings was not recorded neither. Although some problems have been identified with this question, it is still considered to be the best available (Extra and Yagmur, 2010) and most promising indicator for obtaining basic information of the increasingly multicultural societies (van der Merwe and van der Merwe, 2007).

The article "Home language use and shift in Australia: Trends in the new millennium" was published in 2023. Journal: Front Psychol.

### 4.2. Procedures

Using the online facility of TableBuilder provided by ABS, related statistics were derived from the ABS census database step by step. First, to disclose the general situation of people’s home language use and its changing patterns during the past two decades, data regarding the total number of home language users in the whole country and the number of the top ten home languages other than English were collected and analyzed. Comparisons were made between the five data sets after the new millennium. Apart from analyzing the overall situation nationwide, descriptive analyses were also conducted at the regional level to reveal the variations among different states and territories. The proportion of population speaking a home language in different states and territories were calculated based on the data retrieved from the latest five censuses. The top ten home languages other than English and their respective number of speakers in each state and territory were also compared based on the 2021 census. Next, language shift rates of different language communities in the latest available censuses and their cross-tabulations with generations, gender, age, and duration of residence were collected using the TableBuilder again. The data were further compared and arranged manually with the aim to better capture and present the developmental trends.

All the data elicited was subject to comparative analysis. By comparing the population size and ratio of certain groups and calculating the growth rate and the decreasing amplitude of the related data, it is hoped that the general trend of people’s home language use patterns will be clearly presented.

## 5. Results

### 5.1. Home language use in Australia from 2001 to 2021

In the 2021 Australian Census, nine broad groups of languages have been classified based on genetic affinity and the geographic proximity of areas where particular languages originated. Among them are Northern European Languages, Southern European Languages, Eastern European Languages, Southwest and Central Asian Languages, Southern Asian Languages, Southeast Asian Languages, Eastern Asian Languages, Australian Indigenous Languages, and Other Languages. Under the nine broad groups, 51 narrow groups and 494 languages were identified, including 238 Australian Indigenous languages (including 20 not elsewhere classified categories), and 256 non-Indigenous languages (including 24 not elsewhere classified categories). Compared to the 48 Indigenous languages processed in the 1996 census, special attention had been given to identifying more Australian Indigenous languages, for which the criterion for separate identification is three or more speakers.

The article "Home language use and shift in Australia: Trends in the new millennium" was published in 2023. Journal: Front Psychol.

The 2021 statistics showed that of the total population of 25,422,788, there were 5,663,703 people speaking a community language at home, reaching a proportion of 22.3%, which exhibited a 7.2% increase as compared with that in 2001. The sharp increase occurred from 2006 to 2016, with the number of community language users increasing for more than 1.7 million. Among all the community languages, Mandarin has been ranked first by size since 2011. According to the 2021 Census, 685,274 people reported to speak Mandarin in their homes, which account for 2.7% of the total population. The top ten home languages other than English used in Australia in the last four censuses in the past 20 years are shown in Table 1.

**Table 1:** Top 10 community languages in 2021 and the comparison with the previous four censuses.

Year	2021		2016		2011		2006		2001	
Languages	Number of Speakers	Percentage (%)	Number of Speakers	Percentage (%)	Number of Speakers	Percentage (%)	Number of Speakers	Percentage (%)	Number of Speakers	Percentage (%)
**Mandarin**	685,274	2.7 (+0.2)	596,703	2.5 (+0.9)	336,178	1.6 (+0.5)	220,604	1.1 (+0.4)	139,114	0.7
**Arabic**	367,159	1.4 (0)	321,720	1.4 (+0.1)	287,171	1.3 (+0.1)	243,661	1.2 (+0.1)	209,121	1.1
**Vietnamese**	320,758	1.3 (+0.1)	277,391	1.2 (+0.1)	233,388	1.1 (+0.1)	194,854	1.0 (+0.1)	174,027	0.9
**Cantonese**	295,281	1.2 (0)	280,943	1.2 (0)	263,538	1.2 (0)	244,557	1.2 (0)	225,088	1.2
**Punjabi**	239,033	0.9 (+0.3)	132,500	0.6 (+0.3)	71,231	0.3 (+0.2)	23,163	0.1 (0)	14,894	0.1
**Greek**	229,643	0.9 (−0.1)	237,583	1.0 (−0.2)	252,211	1.2 (−0.1)	252,226	1.3 (−0.1)	263,487	1.4
**Italian**	228,042	0.9 (−0.3)	271,602	1.2 (−0.2)	299,829	1.4 (−0.2)	316,894	1.6 (−0.3)	353,229	1.9
**Hindi**	197,132	0.8 (+0.1)	159,637	0.7 (+0.2)	111,349	0.5 (+0.1)	70,006	0.4 (+0.1)	47,766	0.3
**Spanish**	171,370	0.7 (+0.1)	140,813	0.6 (+0.1)	117,493	0.5 (0)	98,002	0.5 (0)	93,410	0.5
**Nepali**	133,068	0.5 (+0.2)	124,010	0.3 (+0.2)	27,156	0.1 (+0.1)	4,654	0	2,497	0
**Total non-English**	5,663,703	22.3 (+1.5)	4,871,647	20.8 (+3.6)	3,912,937	17.2(+2.0)	3,146,195	15.2 (+0.1)	2,853,851	15.1

The number in brackets indicates the change from the previous census.

The article "Home language use and shift in Australia: Trends in the new millennium" was published in 2023. Journal: Front Psychol.

Australian Bureau of Statistics, 2001–2021.

Collectively, Chinese languages, Mandarin and Cantonese together, have the greatest number of speakers after English, accounting for approximately 3.9% of the total population. It is also evident that the number of Chinese speakers, especially Mandarin speakers, has increased steadily over the past 20 years. The number of Mandarin speakers had increased from 139,114 in 2001 to 685,274 in 2021, which is nearly a 5-time increase. Although the percentage of Cantonese speakers among the total population had remained unchanged, the number of its speakers had increased from 225,088 in 2001 to 295,281 in 2021. The steady increase can also be observed in Arabic, Vietnamese, Hindi, Punjabi, and Nepali. Nepali, for the first time, entered the top-10 community language list in 2021. This may well be attributed to the increasing population shares brought by the new arrivers. As the last two decades had witnessed a marked intake of settlers from Asian countries (Ndhlovu and Willoughby, 2017), the percentage of European-born migrants had dropped sharply. The 2021 Census statistics showed that India and mainland China had both overtaken New Zealand to become the second and third country of birth of its oversea population after England, each accounting for 9.6 and 7.8% of the total overseas born, respectively. Skilled migrants from China and other Southeast Asian countries have kept on increasing apace after entering into the new century. At the same time, the number of Arabic speakers, mainly from Lebanon, Iraq, Egypt, etc., was also on a steady increase, making it as the second biggest community language in Australia. On the other hand, languages spoken by the longer established immigrant groups, such as Italian and Greek, were recorded a sharp decrease in the last 20 years. For example, Italian, once the top one LOTE speaking at home, had fallen to the seventh, with its speakers shrinking from 353,229 in 2001 to 228,042 in 2021. Although it is still in the top ten list, it is largely attributed to the huge wave of migrants in the middle of the last century (Clyne and Kipp, 1997; Ndhlovu and Willoughby, 2017). Besides, several other European languages had dropped out the top ten list, such as Yugoslav, German, Polish, and Dutch. It is apparent that many of the well-established European languages have shown a receding trend after entering the new century, and this may be caused by the aging of their populations (Ndhlovu and Willoughby, 2017).

The article "Home language use and shift in Australia: Trends in the new millennium" was published in 2023. Journal: Front Psychol.

In all, the size ranking of the community languages spoken at home has changed considerably during the past 20 years. A more detailed look at the regional differences will be discussed in the next section.

### 5.2. Regional difference of home language speakers of LOTE

When we looked at the home language speakers of LOTE in different states and territories, it can be found that great regional differences were existing. Generally, the numbers of home language speakers of LOTE were on the rise in all the states and territories during the past 20 years. But most of them were inhabiting in New South Wales, Victoria, Queensland, South Australia, and Western Australia. The increases in New South Wales and Victoria were most remarkable, with their home language speakers of LOTE growing from 1,196,204 in 2001 to 2,146,982 in 2021 and 920,820 in 2001 to 1,791,784 in 2021, respectively. The number of home language speakers in the two states had both nearly doubled in the 20 years’ time. Further, when we investigated the data in more details, the picture gets even clearer. Most of these home language speakers in New South Wales and Victoria were settled in two big cities, Sydney and Melbourne. This is the same with the findings of other studies (Clyne and Kipp, 1997; Clyne et al., 2008; Forrest et al., 2020). The concentration rates of the home language speakers of LOTE also presented an upward trend. With 1,727,574 and 1,450,937 home language speakers of LOTE inhabiting in Sydney and Melbourne in 2016 respectively, the numbers had grown by more than 50% as compared with those in 2001. Among these home language speakers, the ones aged between 0 and 14 accounted for around 15% in either Greater Sydney or Greater Melbourne areas. This figure had not changed much in Greater Melbourne; however, in Greater Sydney area, it had dropped by around 2% between 2006 and 2016.

Although the absolute numbers of home language speakers of LOTE were not that big in Queensland and Western Australia, the numbers had been more than doubled as well. Home language speakers in South Australia had grown by 144,810. Tasmania, Northern Territory, and Australian Capital Territory had a relatively slower increase as compared with regions mentioned above, but considering their small base number, the growth rates were glaring as well. Detailed statistics of the number of home language speakers of LOTE for all the states and territories from 2001 to 2021 are presented in Figure 1.

**Figure 1:** Home language speakers of LOTE by state/territory.

The article "Home language use and shift in Australia: Trends in the new millennium" was published in 2023. Journal: Front Psychol.

Besides the increase of the absolute number of home language speakers of LOTE, the proportions of population speaking a community language at home in all regions were on the rise as well. From 2001 to 2021, the ratio of home language speakers of LOTE in New South Wales had increased from 18.77 to 26.60%. Similar trend can also be observed in other states and territories. Nearly all the regions had demonstrated a growth between 5 and 8%. Northern Territory and Australian Capital Territory had exhibited the biggest increase in the past 20 years, whose percentage of home language speakers of LOTE had grown by 10.43 and 11.05%, respectively. Table 2 presents the specific statistics of different regions from 2001 to 2021.

**Table 2:** Proportion (%) of population speaking non-English language at home by state/territory.

	2001	2006	2011	2016	2021
New South Wales	18.77	20.07	22.47	25.16	26.60
Victoria	19.82	20.42	23.07	25.96	27.55
Queensland	6.94	7.76	9.78	11.86	13.22
South Australia	11.76	12.18	14.38	16.35	17.81
Western Australia	11.17	11.58	14.52	17.59	18.39
Tasmania	3.09	3.50	4.47	5.35	8.73
Northern Territory	21.96	23.18	26.74	29.52	32.39
Australian Capital Territory	13.52	14.56	18.10	21.81	24.57

Australia Bureau of Statistics, 2001, 2006, 2011, 2016, 2021 census.

It is evident from the data above that the overall number and the proportion of home language speakers of LOTE were rising in all the regions in Australia. But a closer look at the top ten home languages other than English in each administrative regions further revealed that great regional differences had existed. Languages such as Korean, Filipino, Tagalog, Afrikaans, Japanese, Nepali, Sinhalese, and some Australian Indigenous languages had appeared in different regional lists. The top ten home languages other than English in eight different regions showed similarities as well as differences. Mandarin, as the most wildly used home language nationwide, topped seven regional lists. It was present in all the eight regional lists. Around 72% of Mandarin speakers were in New South Wales and Victoria. Besides, Cantonese and Vietnamese were included in seven regional lists, Italian and Hindi were included in six regional lists. Italian remained to be a stronger home language in New South Wales, Victoria, and Western Australia, the speakers of which in these three states made up for around 80% of its total population. Although its ranking was not very high in New South Wales, the number of Italian speakers there was big as well, only after Victoria, reaching over 64,000. Arabic, though ranked the second in the national list, was absent from the regional lists of Queensland, Tasmania, and the Northern territory. Further looking into the regional statistics, we can find that most of these Arabic speakers were in New South Wales and Victoria, with an outright majority clustered around Sydney. This finding is consistent with Ndhlovu and Willoughby’s study (2017), which also found that Arabic was most widely spoken in Sydney (2.7% of the population). In addition, languages such as Greek, Spanish, and Punjabi were also used widely across at least five regions. And what is particular for the Northern territory is that it was the only state where the Australian Indigenous Languages were included in the top ten home languages. The specific orders and the numbers of home language speakers of LOTE in each region are shown in Table 3.

The article "Home language use and shift in Australia: Trends in the new millennium" was published in 2023. Journal: Front Psychol.

**Table 3:** Top 10 home languages other than English in different states and territories in 2021.

Rank	NSW	VIC	WA	QLD	SA	TAS	NT	ACT
1	Mandarin (270,685)	Mandarin (221,798)	Mandarin (51,751)	Mandarin (83,607)	Mandarin (32,133)	Mandarin (8,129)	Kriol (5,191)	Mandarin (14,397)
2	Arabic (227,243)	Vietnamese (118,801)	Italian (25,432)	Vietnamese (31,370)	Italian (23,828)	Nepali (7,248)	Djambarrpuyngu (3,857)	Nepali (5,859)
3	Cantonese (148,943)	Greek (107,158)	Vietnamese (22,763)	Punjabi (30,873)	Greek (21,882)	Punjabi (2,556)	Greek (3,258)	Vietnamese (5,028)
4	Vietnamese (117,907)	Punjabi (104,949)	Punjabi (20,613)	Spanish (29,642)	Vietnamese (21,855)	Spanish (1,571)	Nepali (3,099)	Punjabi (5,019)
5	Hindi (80,051)	Italian (92,320)	Cantonese (19,683)	Cantonese (27,437)	Punjabi (20,004)	Cantonese (1,536)	Tagalog (3,047)	Hindi (4,769)
6	Greek (78,691)	Arabic (91,441)	Tagalog (17,313)	Korean (21,904)	Arabic (11,003)	Urdu (1,492)	Mandarin (2,526)	Cantonese (4,230)
7	Spanish (71,868)	Cantonese (82,432)	Arabic (16,000)	Hindi (21,344)	Cantonese (10,166)	Vietnamese (1,467)	Warlpiri (2,477)	Spanish (4,122)
8	Nepali (68,148)	Hindi (66,930)	Afrikaans (14,729)	Tagalog (20,603)	Hindi (9,884)	German (1,446)	Filipino (2,101)	Arabic (3,867)
9	Italian (64,039)	Sinhalese (49,501)	Spanish (12,958)	Italian (17,989)	Nepali (9,671)	Hindi (1,284)	Tiwi (2,044)	Urdu (3,638)
10	Korean (62,319)	Spanish (43,181)	FiliPino (12,501)	Japanese (17,928)	Hazaraghi (7,447)	Greek (1,126)	Murrinh Patha (2,044)	Italian (2,816)

The number in brackets indicates the number of speakers.

Australian Bureau of Statistics, 2021 census.

### 5.3. Language shift trend in the new era

With an increasingly diversified immigrant population in the new era, Australian government claimed to have enforced a policy of multiculturalism, which was boasted to help non-English speaking background migrant groups maintain their culture and promote the survival of their community languages within mainstream institutions (Forrest et al., 2020). After analyzing the language data from the 2006 census, Clyne et al. (2008, p. 1) characterized Australia as an increasingly multilingual nation. Some other researchers, however, stated that this is only true for the languages of recently arrived migrants (Forrest et al., 2020). Karidakis and Arunachalam (2016) noted in their study that one in four non-English speaking background children aged 5 or above spoke only English at home. Language shift occurred among different migrant groups with varying degrees. Many factors, such as ancestry place, gender, generation, age, place of residence, level of education, etc., exert certain impact on the language shift trend of different migrant groups (Chiswick and Miller, 1995; Kipp, 2007; Forrest and Dandy, 2017). The following sections will analyze the data relating to the language shift rate of different groups and try to depict a dynamic picture of the language shift patterns of different migrant groups in recent years.

The article "Home language use and shift in Australia: Trends in the new millennium" was published in 2023. Journal: Front Psychol.

#### 5.3.1. Language shift of the first-generation migrants

Language shift of the first generation refers to those who were born outside Australia and spoke a first language other than English now speak only English. Birthplace was used as a surrogate indicator for their language background. Although this may not reflect their language background precisely, especially for those whose home countries are noted for using a diversity of languages, it is proved to be the most feasible and reliable statistical method for calculating language shift rate (Clyne and Kipp, 1997).

Looking at the 2016 data, we can find that the range of the shift rates was further enlarged, extending from 2.63% for those born in mainland China to 65.43% for those born in Netherlands. At the higher end, besides Netherlands, we can also find Germany (53.77%) with a shift rate higher than 50%. At the lower end, there were mainland China (2.63%), Iraq (2.96%), and Vietnamese (3.91%), all with a shift rate lower than 5%. This finding was generally consistent with the patterns found in the previous studies (Clyne and Kipp, 1997; Karidakis and Arunachalam, 2016), showing that those from northern and central Europe usually sustained a higher level of shift rate than those from Asian countries.

Moreover, when we compared the data in 2006, 2011, and 2016, it is evident that the ranking order of the shift rates had changed a lot, but generally, it only fluctuated in a small range with a few exceptions (see Table 4). The most striking variations were concerned with those born in India and Croatia. For those born in India, their language shift rate had declined continuously from 34.41% in 2006 to 21.28% in 2011 and then to 15.62% in 2016, falling from rank 5 to rank 12. On the other side, for Croatia-born community, the ranking position had demonstrated a big increase. Though the absolute value of its language shift rate had only risen for around 3% between 2006 and 2016, from 16.67 to 19.73%, its ranking had risen from number 12 in 2006 to number 7 in 2016. The situation for Serbia-born community was a little different. Its language shift rate had risen from 8.86% in 2006 to 11.00% in 2011 and then to 13.63% in 2016, but its ranking had only moved two places up. On the other side, for the Sri Lanka-born community, although its language shift ranking had only fallen 1 place, the language shift rate had dropped from 34.96% in 2006 to 23.08% in 2016. The similar trend can also be observed on Malaysia-born and Philippine-born communities. The ranking order of these two communities had remained unchanged between 2006 and 2016, however, their language shift rates had dropped from 35.01 to 31.38% and 27.02 to 22.27%, respectively.

The article "Home language use and shift in Australia: Trends in the new millennium" was published in 2023. Journal: Front Psychol.

**Table 4:** Language shift of the first generation by country of birth in 2006, 2011, 2016.

Rank	2006	2011	2016
1	Netherlands (64.41%)	Netherlands (63.71%)	Netherlands (65.43%)
2	Germany (53.89%)	Germany (52.71%)	Germany (53.77%)
3	Malaysia (35.01%)	Malaysia (32.56%)	Malaysia (31.38%)
4	Sri Lanka (34.96%)	Sri Lanka (26.75%)	Poland (24.53%)
5	India (34.41%)	Poland (23.92%)	Sri Lanka (23.08%)
6	Philippines (27.02%)	Philippines (22.64%)	Philippines (22.27%)
7	Poland (23.61%)	India (21.28%)	Croatia (19.73%)
8	Egypt (22.17%)	Egypt (20.26%)	Italy (19.44%)
9	Japan (17.41%)	Italy (17.77%)	Egypt (19.34%)
10	Italy (17.32%)	Croatia (17.55%)	Indonesia (16.84%)
11	Indonesia (17.30%)	Japan (17.44%)	Japan (16.73%)
12	Croatia (16.67)	Indonesia (16.34%)	India (15.62%)
13	Russia Federation (14.14%)	Russia Federation (13.67%)	Russia Federation (14.52%)
14	Hong Kong SAR (11.22%)	Hong Kong SAR (12.48%)	Serbia (13.63%)
15	Korea (10.37%)	Serbia (11.00%)	Hong Kong SAR (12.85%)
16	Serbia (8.86%)	Korea (9.32%)	Turkey (10.30%)
17	Greece (8.56%)	Turkey (8.10%)	Lebanon (8.73%)
18	Turkey (8.15%)	Lebanon (7.41%)	Korea (8.70%)
19	Lebanon (7.40%)	Greece (7.41%)	Greece (8.32%)
20	Iraq (3.88%)	China (excludes SARs and Taiwan) (3.32%)	Vietnamese (3.91%)
21	China (excludes SARs and Taiwan) (3.81%)	Vietnamese (3.23%)	Iraq (2.96%)
22	Vietnamese (2.99%)	Iraq (3.01%)	China (excludes SARs and Taiwan) (2.63%)

The number in brackets indicates the corresponding language shift rate.

Australian Bureau of Statistics, 2006, 2011, 2016 census.

Except the fore-mentioned glaring changes, the variations of language shift rates or ranking orders for other language communities had only demonstrated slight fluctuations. Language shift rates of the following communities, namely, Germany, Egypt, Japan, Indonesia, Korea, Greece, Iraq, and mainland China, had decreased slightly, while others, such as Netherlands, Poland, Italy, Russia Federation, Hong Kong SAR, Turkey, Lebanon, and Vietnamese had risen slightly. The language shift rate variations for these communities were all within 3%, some were even less than 1%. Thus, on the whole, their ranking order remained relatively stable (see Table 4). In all, as observed by previous researchers that the language shift process of different ancestry groups was far from uniform (Forrest et al., 2020).

The article "Home language use and shift in Australia: Trends in the new millennium" was published in 2023. Journal: Front Psychol.

#### 5.3.2. Language shift of the second-generation migrants

Table 5 summarizes the language shift rates of the second generation migrants. Language shift of the second generation refers to those who were born in Australia but with both or one of their parents born overseas and speaking another language other than English now speak only English. Compared with the first-generation migrants, the language shift rates of the second generation were much higher, with the top ten having a shift rate well above 50%. This trend was also found by Clyne and Kipp (2006). For the second generation migrants from Netherlands, which ranked at the top of the list, the language shift rate was as high as around 95%. Even for Vietnamese communities, which ranked last, their second generation language shift rate reached 22.48% in the 2016 census. Further, when we compared the language shift rates of the two generations, the differences were found to be glaring (see Tables 4, 5), with most of the differences between the 1^st^ and the second generation language shift rates larger than 30% (Netherlands, Germany, Malaysia, Indonesia, Egypt, India, Serbia, Greece, China, and Croatia), and some were even larger than 50% (Philippines, Poland, Italy, and Russia Federation).

**Table 5:** Language shift of the second generation by ancestry in 2006, 2011, and 2016.

Rank	2006	2011	2016
1	Netherlands (95.84)	Netherlands (95.11)	Netherlands (94.65%)
2	Germany (91.92%)	Germany (91.17%)	Germany (89.73%)
3	Poland (81.70%)	Poland (81.67%)	Philippines (83.35%)
4	Philippines (79.48%)	Philippines (81.09%)	Poland (82.04%)
5	Russia Federation (75.38%)	Malaysia (74.28%)	Malaysia (75.79%)
6	Malaysia (75.12%)	Russia Federation (72.13%)	Italy (73.46%)
7	Sri Lanka (71.75%)	Italy (71.25%)	Russia Federation (68.94%)
8	Italy (69.59%)	Croatia (64.44%)	Croatia (66.73%)
9	Croatia (61.68%)	Indonesia (58.35%)	Indonesia (59.25%)
10	India (60.90%)	Egypt (55.84%)	Egypt (57.73%)
11	Indonesia (60.16%)	India (53.15%)	India (46.45%)
12	Serbia (59.42%)	Serbia (43.05%)	Serbia (45.51%)
13	Egypt (55.02%)	Greece (41.06%)	Greece (44.78%)
14	Japan (42.16%)	Japan (37.77%)	Sri Lanka (38.97%)
15	Greece (39.17%)	China (37.83%)	China (37.33%)
16	China (37.27%)	Lebanon (30.71%)	Lebanon (37.24%)
17	Lebanon (28.08%)	Sri Lanka (26.69%)	Japan (35.28%)
18	Turkey (21.83%)	Turkey (23.67%)	Turkey (29.54%)
19	Iraq (21.68%)	Korea (20.98%)	Korea (22.69%)
20	Korea (19.24%)	Iraq (20.12%)	Iraq (22.62%)
21	Vietnam (11.29%)	Vietnam (15.45%)	Vietnam (22.48%)

The number in brackets indicates the corresponding language shift rate.

The article "Home language use and shift in Australia: Trends in the new millennium" was published in 2023. Journal: Front Psychol.

Australian Bureau of Statistics, 2006, 2011, 2016 census.

Although the ranking order of the second generation was more or less similar to that of the first generation, slight differences still existed. The ranking differences for most migrant groups were within 3 places, except for Russia Federation, Greece, and China, whose ranking places of the second generation were 5 to 8 places up as compared with that of their first generation. The significant rise of language shift rates in the second generation of these communities was explained by Clyne and Kipp (2006) as reflecting a pragmatic view held by the parents, aiming at providing their children with the best possible access to English and Australian education. The second-generation migrant group from Sri Lanka was another exception, whose language shift ranking was 9 places lower than its first generation in 2016 data set. This may reflect relative successful language maintenance efforts made by the Sri Lanka migrants.

From another perspective, when we compare the statistics from the three censuses (2006, 2011, 2016), it can be found that for most migrant groups the language shift rates of the second generation remained relatively stable, with only a slight fluctuation. The only exception was the shift rate of the second-generation migrants from Sri Lanka, whose language shift rate had plunged from 71.75% in 2006 to 26.69% in 2011, and then raised back to 38.97% in 2016. These particular conditions for Sri Lankan migrants cannot be understood without relating to their homeland political affiliations (Perera, 2015). The civil war in Sri Lanka starting from the 1980s had caused a massive emigration of its people into Australia. With a large increase of Sri Lankan migrants arriving in Australia between 2006 and 2011, most of these new arrivers were more proficient in their community languages than their earlier counterparts (Perera, 2015), and Sri Lankan Australian communities were better established. Similar to the situation of Latvian Australians in the 1940s after the Soviet Union’s takeover of Latvia, passing their languages onto their second or third generation became a priority (Smolicz et al., 2001). They may see themselves as keepers of their cultures in exile. This may lead to their greater language maintenance efforts.

The article "Home language use and shift in Australia: Trends in the new millennium" was published in 2023. Journal: Front Psychol.

#### 5.3.3. Gender and language shift

Analyzing the language shift rate of immigrant communities in relation to gender, we may find that gender differences were not obvious.

For the first generation, the difference of language shift rates caused by gender has always been small, all within the range of −10 to 10% (see Table 6). And the fluctuations of the gender differences for the same birthplace were slight as well. A general trend being observed is that males from most European countries, such as Italy, Netherlands, Croatia, Germany, etc., exhibited a higher language shift rate than females, while females from many Asian countries, such as Philippines, Sri Lanka, Korea, etc., had a higher language shift rate than males. This result is consistent with the findings based on the census statistics of 1986 to 1996 (Holmes, 1993; Clyne and Kipp, 1997; Walker and Heard, 2015). As the previous studies revealed that in more established community groups in Australia, males tended to shift more than females to use English due to a higher exogamy rate among their male members. For the communities from Asian countries, however, the exogamous marriage rates of males were much lower. On the contrary, a large number of women from these cultures moved to Australia in exogamous marriage. Thus, females from these countries demonstrated higher shift rate. But anyhow, the gender difference of language shift rates of communities from Asia was small. The first-generation language shift rates of communities from Iraq, Malaysia, Japan, Vietnam, Hong Kong SAR, India, and mainland China, all displayed a gender difference less than 1% in the 2016 census.

**Table 6:** Difference of the first-generation language shift rate by gender (2006–2016).

	2016			2011			2006		
Birthplace	Male shift rate (%)	Female shift rate (%)	Difference	Male shift rate	Female shift rate	Difference	Male shift rate	Female shift rate	Difference
Italy	24.15	14.53	9.62	22.29	13.04	9.25	21.71	12.61	9.1
Netherlands	69.08	61.71	7.37	67.67	59.60	8.07	68.61	59.98	8.63
Croatia	23.33	16.24	7.09	20.61	14.42	6.19	19.72	13.46	6.26
Germany	57.46	50.48	6.98	56.20	49.54	6.66	57.59	50.48	7.11
Egypt	21.65	16.87	4.78	22.75	17.58	5.17	25.19	19.07	6.12
Greece	10.58	6.24	4.34	9.26	5.64	3.62	10.37	6.78	3.59
Poland	26.96	22.70	4.26	26.72	21.77	4.95	26.59	21.13	5.46
Turkey	12.27	8.20	4.07	9.84	6.24	3.6	9.77	6.42	3.35
Serbia	15.40	11.98	3.42	12.45	9.55	2.9	10.16	7.51	2.65
Lebanon	10.00	7.36	2.64	8.55	6.19	2.36	8.50	6.20	2.30
Iraq	3.42	2.48	0.94	3.62	2.38	1.24	4.57	3.11	1.46
Malaysia	31.46	31.31	0.15	32.62	32.52	0.10	35.39	34.70	0.69
Japan	16.76	16.74	0.02	16.75	17.75	−1.00	15.91	18.15	−2.24
Vietnamese	3.72	4.06	−0.34	3.01	3.41	−0.40	2.89	3.07	−0.18
Hong Kong SAR	12.61	13.08	−0.47	12.39	12.57	−0.18	11.22	11.22	0
India	15.28	16.02	−0.74	20.03	22.85	−2.82	31.28	38.26	−6.98
Mainland China	2.15	3.00	−0.85	2.72	3.80	−1.08	3.26	4.27	−1.01
Indonesia	16.18	17.33	−1.15	15.36	17.13	−1.77	17.17	17.40	−0.23
Russia Federation	13.60	15.04	−1.44	12.62	14.29	−1.67	13.72	14.46	−0.74
Korea	7.77	9.53	−1.76	8.11	10.36	−2.25	9.04	11.48	−2.44
Sri Lanka	22.19	24.05	−1.86	25.99	27.54	−1.55	33.96	35.98	−2.02
Philippines	18.99	24.35	−5.36	18.34	25.25	−6.91	21.64	29.96	−8.32

Australian Bureau of Statistics, 2006, 2011, 2016 census.

The article "Home language use and shift in Australia: Trends in the new millennium" was published in 2023. Journal: Front Psychol.

Further, by analyzing the data from the past censuses, it was found that great variations occurred among communities from Japan, India, and Philippines. The difference of male/female language shift rate for the first-generation migrants from Japan was reported to be −4.7% in 1996 (Clyne and Kipp, 1997), however, this difference was narrowed down to −2.24% in 2006, −1% in 2011 and further down to 0.02% in 2016. Similar trend can also be found for the first-generation migrants from India (−6.98% in 2006 to −2.82% in 2011 and down to −0.74 in 2016) and Philippines (−8.32% in 2006 to −6.91% in 2011 and down to −5.36% in 2016). This narrowing trend may be resulted from the ever-increasing number of community language speakers since the new millennium. The imbalance between the number of male and female migrants from these community groups tend to be reduced. As Clyne and Kipp (1997, p. 466) argued that where there is a larger number of men or women in the community, they may be expected to display a higher language shift rate. The reduced male/female variation in language shift may well be caused by the change of the sex ratio of these community groups.

When it comes to the second generation, the gender differences were further reduced. In all the three census statistics (2006, 2011, and 2016), the gaps between male and female for all migrant communities were kept under 2%. This is consistent with the findings based on the previous census statistics (Clyne and Kipp, 1997). As is explained by Clyne and Kipp (1997), this may be due to the fact that the influencing factors working for the first generation were no longer effective for the second generation.

#### 5.3.4. Age and language shift

Based on the 2016 census data, age-related difference in language shift rate of the first-generation migrants demonstrated great variations for different migrant groups (see Table 7). Similar to the previous findings (Clyne, 1991; Clyne and Kipp, 1997), several migrant groups showed the lowest shift rates among their oldest groups (+65-year-olds), notably among Turkish, Lebanese, Korean, Greece, and Vietnamese Australians, while in some other migrant groups, it was their youngest children (0-4-year-olds) who shifted least. The communities with the youngest group featuring the lowest shift rate were generally those coming from European countries, including Netherlands, Germany, Poland, Croatia, Egypt, and Russia Federation. Besides, Japan was also one of them. For other community groups, however, the ones who shifted least showed a dispersed tendency across all age groups. Some with their 15-24-year-olds shifted least (Malaysia, Serbia, and mainland China), some with 25–34-year-olds shifted least (Italy, Indonesia, and India), still, others with their 35–44-year-olds (Sri Lanka, Iraq) or 45–54-year-olds (Philippines), or 55–64-year-olds (Hong Kong SAR) shifted least.

The article "Home language use and shift in Australia: Trends in the new millennium" was published in 2023. Journal: Front Psychol.

**Table 7:** Language shift rate by age in the first generation.

Rank	2016	0–4	5–14	15–24	25–34	35–44	45–54	55–64	+65
1	Netherlands (65.43%)	24.74	37.45	41.87	37.64	45.71	55.45	77.26	69.61
2	Germany (53.77%)	21.24	29.70	27.81	35.30	36.78	49.83	65.42	61.06
3	Malaysia (31.38%)	28.01	37.61	23.68	27.58	31.97	38.75	34.83	31.49
4	Poland (24.53%)	12.35	15.81	15.44	24.02	28.24	20.80	19.82	27.75
5	Sri Lanka (23.08%)	21.88	21.50	19.94	16.47	13.67	20.82	31.78	46.60
6	Philippines (22.27%)	45	35.23	24.29	25.10	18.56	17.20	21.59	20.01
7	Croatia (19.73%)	0	18.58	10.86	14.30	16.73	32.92	23.21	15.53
8	Italy (19.44%)	14.59	15.26	13.27	12.85	18.90	36.25	34.63	14.67
9	Egypt (19.34%)	8.5	14.69	11.81	11.45	8.61	17.82	22.89	26.36
10	Indonesia (16.84%)	24.85	23	13.46	12.35	14.79	16.49	21.09	30.42
11	Japan (16.73%)	9.41	18.31	23.32	18	11.06	14.78	22.03	25.50
12	India (15.62%)	18.62	14.79	14.26	7.56	8.85	25.97	36.03	57.46
13	Russia Federation (14.52%)	4.3	7.52	16.25	18.58	12.83	13.56	10.75	15.81
14	Serbia (13.63%)	10	6.66	5.62	15.24	14.42	21.04	7.99	10.23
15	Hong Kong SAR (12.85%)	25.57	40.47	12.36	11.40	13.97	13.31	8.27	11.62
16	Turkey (10.30%)	13.27	14.65	10.43	11.23	10.63	12.70	8.91	5.95
17	Lebanon (8.73%)	11.14	14.05	6.96	7.24	8.67	11.83	7.75	6.94
18	Korea (8.70%)	6.15	15.29	10.68	12.38	6.46	5.23	3.64	2.40
19	Greece (8.32%)	9.27	5.94	8.80	12.96	12.75	20.70	16.71	4.44
20	Vietnamese (3.91%)	7.65	6.81	3.33	4.30	7.69	2.74	1.55	1.49
21	Iraq (2.96%)	4.98	3.91	2.64	3.23	2.22	2.54	3.37	3.74
22	Mainland China (2.63%)	4.64	7.88	1.80	2.28	2.19	2.40	2.30	4.85

Australian Bureau of Statistics, 2006, 2011, 2016 census.

On the other side, for the age groups which demonstrated the highest shift rates within their communities, three major variations can be observed. Migrant groups with their overall language shift rates at the higher end mostly showed a tendency of older age groups shifted most, 55–64-year-olds (Netherlands, Germany) or + 65-year-olds (Sri Lanka, Egypt, Indonesia, Japan, India), while migrants groups with their overall language shift rates at the lower end mostly showed a tendency of younger age groups shifted most, 5-14-year-olds (Hong Kong SAR, Turkey, Lebanon, Korea, and mainland China) or 0-4-year-olds (Iraq). Other migrant communities were with their highest language shift rates occurred in the middle-aged groups, 25-34-year-olds (Russia Federation), 35-44-year-olds (Poland, Vietnam), or 45-54-year-olds (Malaysia, Croatia, Italy, Serbia, and Greece).

The article "Home language use and shift in Australia: Trends in the new millennium" was published in 2023. Journal: Front Psychol.

So overall it is hard to say which age groups were likely to shift most or least among the first-generation migrants. Different migrant communities showed a different feature. These differences may be caused by their overall community language shift trends, population of different age groups, family language policy and a range of other factors. In all, the bipolarity state of language shift observed by previous researchers (Clyne and Kipp, 1997) has been weakened.

As to the second generation, the shift patterns of different communities seemed to be more consistent than those of the first generation. It is generally the youngest pre-school children who shifted least, and there is a tendency of middle-aged group (35-44-year-olds) or older group (55-64-year-old) shifted most. With the increase of age, their language shift rates rose gradually till 35-44-year-old or 55-64-year-old. The big increases for the second-generation children from communities with higher shifting rates usually occurred around school age group (5–14 years old) or teens to twenties group (15–24 years old) and then slowed down, sometimes with slight decline. It is apparent that these children were likely to shift to use English at an earlier age. On the other side, for those with overall shifting rates at the lower end, the shifting patterns of their second-generation children demonstrated a slow increase in early years. The most glaring increases usually occurred in their middle-aged groups (25–34 or 35–44 years old). The second generation of Vietnamese, Iraq, Korean, and Chinese ancestry all confirmed this trend.

#### 5.3.5. Residence duration and language shift

Table 8 gives us a snapshot about the language shift rates by arrival time based on 2016 statistics. A general trend observed is that for most groups, the language shift rates dropped as their arrival time close to present. Comparing the statistics of the two periods of arrivals, 1986–1995 and 2006–2015, we found that the groups with a difference above 10 % include migrant groups from Netherlands, Germany, Malaysia, Sri Lanka, Philippines, and India, which were all among the top half of the higher language shift groups. Among them, migrants from India exhibited the biggest difference, dropping from 37.62% in 1986–1995 arrivals to 7.59% in 2006–2015 arrivals. This might reflect a fact that migrants from these groups were more likely to shift to use English with their stay in Australia extending. This may as well be due to a range of other factors relating to their linguistic background, marital status, career development, community relations, heritage language programs, etc. In case of Indian-born population, the sharp increase of migrants between 2004 and 2009, which had been nearly doubled, might constitute a major reason. Besides the above-mentioned groups, language shift rates of five other migrant groups also demonstrated an obvious downward trend, with a decline between the two periods above 5%. These include Italy, Indonesia, Serbia, Korea, and Greece.

The article "Home language use and shift in Australia: Trends in the new millennium" was published in 2023. Journal: Front Psychol.

**Table 8:** Language shift rates by residence duration.

Birthplace	Arrived 1986–1995	Arrived 1996–2005	Arrived 2006–2015	Difference between 1986–1995 and 2006–2015
Netherlands (65.43%)	54.56	40.64	27.16	−27.4
Germany (53.77%)	43.56	29.91	27.96	−15.6
Malaysia (31.38%)	33.44	27.70	20.34	−13.1
Poland (24.53%)	17.81	16.36	16.24	−1.57
Sri Lanka (23.08%)	27.20	14.44	9.02	−18.18
Philippines (22.27%)	29.55	25.46	14.17	−15.38
Croatia (19.73%)	13.26	5.86	10.32	−2.94
Italy (19.44%)	19.57	16.50	10.42	−9.15
Egypt (19.34%)	10.69	10.75	6.25	−4.44
Indonesia (16.84%)	18.49	14.65	10.57	−7.92
Japan (16.73%)	18.05	14.88	13.23	−4.82
India (15.62%)	37.62	16.97	7.59	−30.03
Russia Federation (14.52%)	14.26	14.68	10.44	−3.82
Serbia (13.63%)	12.02	6.77	6.21	−5.81
Hong Kong SAR (12.85%)	7.72	12.33	11.74	4.02
Turkey (10.30%)	8.03	7.68	9.72	1.69
Lebanon (8.73%)	6.25	5.15	4.18	−2.07
Korea (8.70%)	13.57	8.65	5.95	−7.62
Greece (8.32%)	11.58	13.40	4.37	−7.21
Vietnamese (3.91%)	2.18	2.99	3.06	0.88
Iraq (2.96%)	4.90	2.56	1.54	−3.36
China (excludes SARs and Taiwan) (2.63%)	3.59	2.67	1.69	−1.9

Australian Bureau of Statistics, 2006, 2011, 2016 census.

However, in Table 8, we can also find a reverse trend. Language shift rates of three groups, migrants from Hong Kong SAR, Turkey, and Vietnam, were on a slight rise. The increase demonstrated by migrants from Hong Kong SAR was the biggest, rising from 7.72% among 1986–1995 arrivals to 11.74% among 2006–2015 arrivals. This is contradictory to the previous trend found by Clyne and Kipp (1997) based on the 1996 statistics, in which language shift rate of migrants from Hong Kong SAR showed a gentle decline as their arrival time drawing near. The higher language shift rate by the newly arrivals from Hong Kong SAR in recent years may be explained by the change of population composition of the migrant group. As the Australia’s immigrant policy shifted to favor more skilled and business immigrants from the emerging Asian economic centers, the newly arrived migrants were generally with a higher level of tertiary education. And many of them obtained their university qualification in Australia. So, as Clyne and Kipp (1997) commented, this may attitudinally and socially promote a shift to English.

The article "Home language use and shift in Australia: Trends in the new millennium" was published in 2023. Journal: Front Psychol.

## 6. Discussion

Language shift is a complicated social phenomenon influenced by a number of variables, including language policies, the concentration of migrant speakers, generations, migrants’ marriage patterns, economic and trade ties between the host country and the migrants’ ancestry countries, etc. Statistics from the censuses in the past 20 years showed that the number of community language speakers in Australia has soared up quickly and great variations have been found between the traditional European migrant groups and the newly Asian arrivers. While the well-established European language communities, such as Italian and Greek, shank remarkably, several Asian languages, such as Chinese, Vietnamese, and Hindi, demonstrated a big increase in its speakers. This changing trend cannot be understood alone without considering a range of social, economic, and political factors.

### 6.1. The changing demographic composition of migrant groups and the changing population speaking a LOTE at home

Australia is a traditional migrant country. Anglo- and Euro-centric migrants had made up for a major part of the Australian immigrant population till the 1980s. Over the past 30 years, however, Australia’s immigration policy has shifted from a focus on family reunion to skills-based migration, which has resulted in the intake of a more diverse migration population (Chik, 2019). Under such a circumstance, the fastest growing demographic groups from Asia and Middle East, have led several languages, including Chinese and Arabic, to rise to the top list of community languages at either national or regional levels. Chinese Mandarin has seized an absolute predominance. On the other side, the languages of postwar European migrants, such as Greek and Italian, have demonstrated constant declining shares among the non-English speaking population. It cannot be denied that the changing order of the community languages is a manifestation of the changing immigration policy and population in Australia, which in turn may point to the changing demand of the LOTE education in the future. How to accommodate the language needs of the increasingly diverse population today becomes a big challenge facing the Australian government. Given the complex picture of their linguistic background, a true multicultural education which cares not only the language needs of the well-established communities but also the new arrivers should be implemented. Due attention should also be paid to the teaching of both English and LOTE so as to help them adapt to the mainstream society easily while maintaining their heritage language as well. Besides, it also needs to be recognized that under the impact of learning technologies, global media, and transnational networks, the teaching requirements of the community languages may change a lot. The focus of the LOTE education should thus not be confined to the provision of different languages in the repertoire, but also care the changing demands and language levels of the migrant population.

The article "Home language use and shift in Australia: Trends in the new millennium" was published in 2023. Journal: Front Psychol.

Moreover, the uneven distribution of the migrant population across the country may also raise different language demands. In areas where the traditional European migrants concentrated, more language service supports may need to be provided for the aging, while in the areas where most new arrivers gathered, providing high-quality multicultural education helping their younger generations maintain their language heritage is important. Anyhow, as Chik (2019) maintained migrants brought languages, and the diverse migration population made Australia a more culturally and linguistically complex society.

### 6.2. Potential factors impacting the language shift

Kalantzis et al. (1989) once commented the position and survival of languages within a multicultural society are closely associated with power relations, self-determination, and access. This is indeed true in an age when the world becomes increasingly globalized and interconnected. The transformative social, political as well as economic agents in the new century may all contribute the migrants’ language choice in the new era.

#### 6.2.1. The growing economic strength of Asian powers

The socio-economic progress of migrants’ ancestries may have a significant impact on their language use patterns (Chiswick et al., 2004; Karidakis and Arunachalam, 2016). The strong momentum of the Asian economy from the beginning of the 21^st^ century has inevitably invigorated the promotion of Asian languages and cultures worldwide. According to the report published by the Australian Department of Foreign Affairs and Trade (DFAT), seven Asian countries, including China, Japan, Republic of Korea, Singapore, India, Malaysia, and Thailand were among Australia’s top ten two-way trading partners (DFAT, 2020). Other relevant statistics, in particular those pertaining to China-Australia economic and trade cooperation, also reveal that the volume of their bilateral trade has climbed from less than $100 million since the two countries established diplomatic relations in 1972 to more than $230 billion in 2021. China has become Australia’s biggest trading partner, export market, import supplier, source of international students, etc. (DHA, 2020, 2022). With the core of Australia’s international trade being relocated to the Asia-Pacific region, the status of these Asian community languages has surely risen in society. Besides, the closer economic ties between Australia and these Asian countries might further boost migration movement to Australia, bringing new vitality to the development and use of these community languages. In the foreseeable future, the growing interests in Asian languages are predeterminate.

The article "Home language use and shift in Australia: Trends in the new millennium" was published in 2023. Journal: Front Psychol.

#### 6.2.2. Favorable policies for community language maintenance

Language policy and planning (LPP) has always been considered as an important factor for language maintenance (Hornberger and Coronel-Molina, 2004; Liddicoat, 2018). With an increasingly economic character prevailing, the previously marginalized voices calling for Australian accommodation to its Asian geographic and security context had transformed into the dominant language interests (Anderson, 2012). The historical preference for European languages has gradually been replaced by the recent preference for community languages, especially for a few selected Asian foreign languages. Policies concerning the protection of the community languages and provisions allowing for the establishment of ethnic schools and organizations have collectively fueled up community language use (Karidakis and Arunachalam, 2016). “Maintenance and development of LOTE” and “provision of services in LOTE” have been emphasized in the *National Policy on Languages.* Nine languages, including Arabic, Chinese and Japanese, have been prioritized for instruction. In Australia’s 1994 *National Asian Languages and Studies in Australian Schools Strategy*, the study of the four Asian languages, namely, Chinese, Japanese, Indonesian and Korean, has received unprecedented attention. And in the first decade of the 21st century, the Australian government has further increased its support for Asian languages with the promulgation of the *National Asian Languages and Studies in School Program*, which had allotted 62.4 million Australian dollars to support students’ learning of Asian languages. Meanwhile, the well-established “ethnic infrastructure” in the long-standing migrant communities (Chiswick et al., 2001; Hugo, 2011; Karidakis and Arunachalam, 2016), and migrants’ easier access to Internet, community radio, and television (Rubino, 2010) would also facilitate the maintenance of their community languages. In 2020, approximately 783 community language schools were in operation in Australia, instructing 105,350 students learning 93 languages, predominantly in NSW and VIC (AFESA, 2021).

The article "Home language use and shift in Australia: Trends in the new millennium" was published in 2023. Journal: Front Psychol.

In brief, it is obvious that the recent favorable language policies for community languages, especially for certain Asian languages, have played an indispensable role in encouraging migrants to maintain and develop their community languages. How far could the favorable policies be executed toward the community languages in a long run may act as a compass in the language life of migrants.

#### 6.2.3. Culture distance to the ancestry

From a macro perspective, the process of language shift is far from uniform (Forrest et al., 2020). Kipp et al. (1995) once argued that migrants’ perceptions of their homeland culture and the ties they had with their ancestries may contribute a lot to the maintenance of their heritage languages. In the previous analysis in this paper, it is not hard to find that either for the first or the second generation, migrants from Anglo- ancestries, such as Netherlands and Germany, demonstrated a much higher language shift rates than those from Asian countries. This can be attributed to a number of cultural and linguistic factors. Among them, a higher level of exogamy in European migrants is one major reason that cannot be neglected. For the newly arrivers from Asia, however, the glaring culture distance caused by different language families, religions, lifestyles, value, etc. may become a hindrance for them to shift to use the new language in the host country. Culture distance can also explain the sharp increase of the language shift rate among the second generation migrant groups. A loose tie to their home country and the shortened distance to the host country both contribute to their higher language shift rates. The “Core value” theory proposed by Smolicz (1981) was often adopted by previous researchers to explain migrant groups’ language shift or maintenance behavior. The relatively lower language shift rates of Greek, Mandarin, Turkish, etc. communities in the present study can be seen as perfect evidence. In this respect, as the proportion of the skilled and professional migrants keeps on increasing in Australia in the new century, there might be a more positive social attitude toward the retention of the languages and cultures brought by the new migrants, which, in turn, may also help later generations to establish a closer linkage to their ethnic identity and maintain a closer tie with their home countries. The future for Australia as a multilingual society can be seen through the ways people connect themselves with their homeland culture.

The article "Home language use and shift in Australia: Trends in the new millennium" was published in 2023. Journal: Front Psychol.

## 7. Conclusion

According to the census statistics from the last 20 years, we can find that the total number of home language speakers of LOTE was on a steady increase. In the 2021 census, this number had reached over 5.6 million, accounting for 22.3% of the total population. As was expected by Clyne and Kipp (1997) and Clyne et al. (2008), Mandarin, Arabic, Cantonese, and Vietnamese had displaced Italian and Geek, becoming the most widely used community languages in Australia. Specifically, the growth rate of Mandarin speakers was surprising. In just a decade, from 2006 to 2016, the number of Mandarin speakers had grown by 170%, overtaking Arabic in 2011 and topped the list since then. Further, the falling trend of German speakers as predicted by Clyne and Kipp (1997) had also been confirmed. According to the latest data, German had fallen out of the top ten community languages in 2016. Regional differences, however, had also existed. Mandarin had seized an overwhelming position, topping the lists of seven states and territories. New South Wales and Victoria had remained to be the two major places that had the most home language speakers of LOTE. The results of the present study showed a positive trend of home language maintenance in the current Australian society.

The changing order of the home languages other than English in the past 20 years may well reflect the changing composition of Australia’s migrant population. It can not only help us to better understand the language needs of an increasingly diverse Australian society but also determine the key factors in predicting the language shift and maintenance trends in the future. The great variations of language shift rate in different communities may be related to a range of sociocultural, linguistic, economic, and political factors. Among them, cultural distance, ethnolinguistic vitality, population concentration, and community dynamics all exert nonnegligible influence (Clyne and Kipp, 1997; Chiswick et al., 2001). Although as Piller (2016) once commented English, the ‘hyper-central language of globalization’, would wash away other languages introduced into Australian society after a few generations, the multicultural policies promoted by the Australian government in recent years did contribute to the increasing number of home language speakers of LOTE. To further maintain the rich linguistic resources in Australia, the government still needs to step up its effort to support community languages in the school system.

The article "Home language use and shift in Australia: Trends in the new millennium" was published in 2023. Journal: Front Psychol.

Anyhow, as Clyne and Kipp (1997) commented that while some community languages declined substantially, other newer ones emerged and rose significantly. And that is the multilingual Australia today with an ever-changing profile of linguistic and cultural diversity.

## Data availability statement

The original contributions presented in the study are included in the article/supplementary material, further inquiries can be directed to the corresponding author.

## Author contributions

LZ contributed to the design of the study, analysis of the data, and writing of the first draft. LT contributed to the conception of the study and the analysis of the data. XQ wrote sections of the manuscript. All authors contributed to the manuscript revision and read and approved the submitted version.

## Funding

The work was supported by the National Social Science Fund of China, grant number: 22XYY027.

## Conflict of interest

The authors declare that the research was conducted in the absence of any commercial or financial relationships that could be construed as a potential conflict of interest.

## Publisher’s note

All claims expressed in this article are solely those of the authors and do not necessarily represent those of their affiliated organizations, or those of the publisher, the editors and the reviewers. Any product that may be evaluated in this article, or claim that may be made by its manufacturer, is not guaranteed or endorsed by the publisher.
